# Adverse Reaction of Acupuncture and Antihypertensive Drugs for Treatment of Essential hypertension: A Protocol for Bayesian Network Meta-Analysis

**DOI:** 10.1155/2022/7397307

**Published:** 2022-08-21

**Authors:** Jiawei Han, Jiwei Yang, Yuanhao Du

**Affiliations:** ^1^First Teaching Hospital of Tianjin University of Traditional Chinese Medicine, Acupuncture Department, Tianjin 300381, China; ^2^Institution of Acupuncture and Moxibustion, China Academy of Traditional Medical Science, Beijing 100700, China

## Abstract

**Background:**

Hypertension, as a high risk factor of cardiovascular disease, has led to a significant upward trend in the population and incidence of the disease. Hypertension patients need to take antihypertensive drugs for life, and therefore people gradually pay more attention to the adverse reactions of antihypertensive drugs. This study protocol outlines a plan to assess the adverse reaction of the different antihypertensive drugs and acupuncture in order for clinical application.

**Objective:**

To compare the side effects of different antihypertensive drugs and acupuncture in the treatment of hypertension.

**Methods:**

and analysis. We will search the databases containing CNKI, Wan-Fang database, Chinese Scientific Journal Database(VIP), PubMed, Cochrane, and Embase, and randomized controlled trials (RCTs) of commonly used antihypertensive drugs or acupuncture for primary hypertension will be obtained. Then, Stata14.0 and Gemtc will be used to assess the statistics. *Ethics and dissemination*. Since no personal patient consent will be required in the study, there is no ethical approval. The results of this reporting will be submitted to a peer-reviewed publication. PROSPERO registration number: CRD42020152703.

## 1. Introduction

### 1.1. Description of the Condition

Hypertension has become a huge challenge to global public health. In recent years, evidence-based medicine has proved that controlling blood pressure can effectively reduce the risk of cardiovascular and cerebrovascular diseases [1]. Decreasing systolic blood pressure by 10–12 mmHg and diastolic blood pressure by 5-6 mmHg can reduce the risk of stroke by 40%, the risk of coronary heart disease by 16%, and the total mortality rate reduce by 20%. If the disease is not treated in time, it can lead to cardiovascular events and seriously threatens the patients' health and quality of life. Effective treatment of hypertension can improve patients' blood pressure and prognosis [2]. It is an important and dangerous cause of many kinds of cardiovascular and cerebrovascular diseases. Although a variety of antihypertensive drugs have been proved to be effective in lowering blood pressure, the low rate of blood pressure controlled by drug therapy is common worldwide [3]. Different patients may have different reactions to the same drug. There are many factors affecting the antihypertensive response of drugs, including age, sex, weight, blood pressure level before treatment, risk factors for combined medication, target organ damage, and drug quality [4]. At present, the most commonly used treatment of hypertension is drug therapy. Since the life-long use of antihypertensive drugs inevitably causes liver and kidney damage, we can consider the feasibility of traditional Chinese medicine in the treatment of hypertension, in which acupuncture is simple and easy to operate, safe and reliable, suitable for personalized treatment, and has unique advantages such as two-way benign regulation and a moderate range of blood pressure reduction, suitable for a large number of people in the early stage of hypertension [5]. It is widely used in clinical practice.

### 1.2. Description of the Intervention

Acupuncture is one of the treasures of traditional Chinese medicine (TCM). It is a subject guided by the theory of TCM to explore the use of acupuncture to prevent and treat patients' diseases. Because of its complexity, it emphasizes the combination of theory and practice. After thousands of years of development, especially through the improvement and promotion of modern Chinese medicine experts, the knowledge system of acupuncture has become increasingly rich and perfect [6]. It is an important part of the theoretical system of TCM with unique academic characteristics, including meridian and acupoints, acupuncture method and the treatment of clinical diseases. In addition, it has a significant therapeutic effect on the nervous system and other diseases.

In general, the commonly used anti-hypertensive drugs in the clinic mainly include angiotensin receptor blocker (ARB), diuretics, *β* receptor blockers, angiotensin converting enzyme inhibitor (ACEI), and calcium channel blockers (CCB). Due to the significant diversity in physical conditions, especially in the elderly, there must be different grades of decline in drug metabolism and excretion function of the liver and kidney [7, 8]. Biochemical monitoring can identify potential adverse reactions during antihypertensive administration [9]. There are many factors that affect the biological availability and distribution of drugs, such as the number of plasma proteins bound by drugs, the volume of circulating plasma, and the proportion of adipose tissue. [10] The physiological changes affected by pharmacokinetics, as well as clinical complexity, and combined medication resistance are all considered to be increased risk of adverse reactions in the elderly [11]. So patients will have different degrees of reactions after taking drugs, and the adverse reactions of anti-hypertensive drugs are significantly various.

### 1.3. Strengths and Limitations of this Study

- This study will include more types of hypertension drugs than before, in addition, nonpharmacotherapy, and acupuncture, will also be taken into account
- The quality of evidence will be assessed by the Grading of Recommendations Assessment, Development, and Evaluation system
- Our research method will focus on types of interventions, but regardless of the dosage, acupoint selection, and acupuncture manipulation
- RCTs that we will retrieve are from English and Chinese databases, which could lead to language bias

## 2. Objectives

The objective of this network meta-analysis is to compare the side effects of different antihypertensive drugs and acupuncture in the treatment of hypertension.

## 3. Methods

The study protocol has been registered on PROSPERO (registration number: CRD42020152703). Our research will comply with the Cochrane Collaboration Handbook [12] and the Preferred Reporting Items for Systematic Reviews and Meta-Analyses Protocols statement (PRISMA-P). [13].

## 4. Eligibility Criteria

### 4.1. Types of Studies

The clinical trials are all randomized controlled trials about acupuncture or common antihypertensive drugs for the treatment of hypertension, the original literature of animal experiment, academic conference, review, and republished literature will be excluded. There are only papers published in Chinese or English.

### 4.2. Types of Participants

The subjects meet the diagnostic criteria of Prevention, Detection, Evaluation, and Management of High Blood Pressure in Adults [14] or any other generally acknowledged diagnostic guidelines. And, they are diagnosed as patients(≥18 years old) with essential hypertension.

### 4.3. Types of Interventions

The intervention measures of the experimental group and the control group are (1) acupuncture: manual acupuncture (MA), electroacupuncture (EA), fire needle (FN), and warm needling moxibustion (WNM); (2) ACEI: benazepril, enalapril, fosinopril, ramipril, and captopril; (3) ARB: valsartan, telmisartan, and losartan; (4) *β* receptor blockers: atenolol, bisoprolol; (5) CCB: amlodipine, levamlodipine, nifedipine, nifedipine controlled release, nifedipine sustained release, nitrendipine, indapamide, felodipine, verapamil, diltiazem, and diltiazem extended release; (6) diuretics: hydrochlorothiazide (HCTZ). In order to clearly compare the adverse reactions of each treatment, we excluded the combination of drugs.

### 4.4. Outcome

We will only record the number of side effect events related to acupuncture or antihypertensive drugs as the primary outcome, and the secondary result is the frequency of each side effect reaction.

### 4.5. Search Strategy

To collect the RCT of acupuncture treatment for essential hypertension, We will search the following electronic databases: China National Knowledge Infrastructure (CNKI), Wanfang Database, China Biology Medicine Database (CBM), EMBASE, PubMed, the Cochrane Central Register of Controlled Trials, at the same time, gray documents such as dissertations and conference papers are also within the scope of retrieval. In addition, consulting references of included studies to supplement the relevant literature. Search is based on the combination of medical subject headings terms and entry terms and the search date is from the establishment of databases to September 1, 2019. The search strategy of PubMed is as follows (Table 1).

## 5. Study Selection and Data Extraction

Studies from the database will be managed by EndNote X9 software to remove duplicate articles.

According to the inclusion and exclusion criteria, two researchers read the topics and abstracts for screening, and then search and read the full text for rescreening. If they have different opinions, a third researcher will assist in solving the problem.

The process of including and excluding studies will be shown using the PRISMA flow chart (Figure 1) [13].

Data are extracted using a unified Microsoft Excel 2007, which included (1) the basic information included in the study: research topic, first author's name, and publication year; (2) the baseline characteristics of the subjects: sample size, age, and gender of patients in each group; (3) intervention measures: drug type, dose, frequency, and course of treatment. (4) Relevant factors of biased risk assessment: random methods, allocation concealment, blind methods, integrity of outcome data, selective reporting of research results, and followup; (5) Outcome indicators: the total number of adverse reactions in each group and the number of events for any one of adverse reactions.

### 5.1. Quality Assessment

Inclusive studies will be evaluated by two researchers using the bias risk assessment tool recommended in Cochrane Cochrane Manual 5.1 [15]. It consists of six aspects: selection bias, performance bias, measurement bias, followup bias, reporting bias, and other biases. The quality of evidence for the included studies will be evaluated by the Grading of Recommendations Assessment, Development, and Evaluation System (GRADE), [16] which contains 4 levels: very low level, low level, moderate level, and high level.

### 5.2. Conventional Meta-Analyses

We will use Stata14.0 software for the statistical analysis of data. *Q* statistics, *I*^2^, and Galbraith diagrams will be conducted to evaluate clinical and methodological heterogeneity test. *I*^2^ ≤ 50% suggest that there is no or slight heterogeneity among the researches and a fixed effect model will be used. [17] If *I*^2^＞50% and the source of heterogeneity would be found, we also present a subgroup analysis. Revman 5.3 software and funnel plot will be conducted to assess publication bias risk. According to Cochrane Risk Bias Assessment Tool, bias risk diagrams are like traffic lights in bias risk images, red represents high risk, yellow represents unclear risk, and green represents low risk. We make use of relative risk (RR) and 95% confidence interval (95% CI) as effect analysis statistics. In order to ensure the accuracy of the conclusions, we will conduct a sensitivity analysis to exclude the literature with nonstandard research methods.

### 5.3. Network Meta-Analyses

Statistical analysis is performed by Stata14.0 and Gemtc software. The triarm experiments will be first divided into two-arm experiments, the adverse reaction rate (relative risk, RR) is used as the amount of effect, and 95% credible interval (95%CrI) of RR is calculated. If the number of occurrence in the analysis data is 0, it is corrected by 1. The network plot and funnel plot will be made by Stata14.0 software, and the funnel plot will be made to monitor the existence of publication bias or small sample effect. The consistency test is conducted by Gemtc software. According to the prior probability, the posteriori probability is inferred. The Bayesian inference is performed by using Markov chain Monte Carlo (MCMC). The fixed effect model is adopted to set the number of iterations as 400000 and the number of annealing as 50000 to eliminate the influence of the initial value. Four chains will be used to simulate and observe the convergence degree. The relationship between interventions is presented by a network graph. Furthermore, the ranking diagram will be produced to sequence the probabilities of an optimal intervention.

## 6. Discussion and Conclusions

Hypertension is an important global public health challenge, as an important risk factor for cardiovascular disease, it is estimated to be the leading cause of death worldwide by 2020 [18]. Affected by the aging population in China, people over 60 and over 80 will account for 29.7% and 7.6% of the total population of China, respectively, by 2050 [19]. Hypertension has a far-reaching impact on disease prevention and public health in the elderly. Considering the economic costs associated with hypertension, early detection and proper blood pressure control are essential to avoid long-term complications of hypertension [20]. Drug therapy is an important means to control the development of hypertension, and drug compliance is the key to achieve the expected clinical efficacy. Foreign studies have reported a significant correlation between adherence to medication and blood pressure control. Studies have reported a significant correlation between adherence to medication and blood pressure control [21, 22]. At present, more and more studies have found that medication compliance of hypertensive patients is related to a variety of physical and mental factors, including depression, poor social support, poor quality of life, and psychosocial factors, which have a great impact on the maintenance of adherence to medication in the elderly [23].

There is a certain objective material basis for acupuncture in the treatment of hypertension. It is related to the effects of nervous system regulation, hemodynamics, cardiovascular activity and humoral regulation etc., which shows that acupuncture treatment of hypertension has the characteristics of multichannel and multitarget [24, 25]. It is suggested that acupuncture may play a role in reducing blood pressure by regulating the neurohumoral-endocrine system through the meridian system [26, 27]. However, through reading a large number of literature, it is found that there are still many deficiencies in the related research of acupuncture treatment of hypertension; for example, the lack of long-term followup of patients in clinical research leads to the lack of evidence for the long-term efficacy of acupuncture treatment of hypertension; it is difficult to achieve blind method in clinical acupuncture treatment, the experimental design is not rigorous enough, and there is no unified clinical path into the standard. To solve the above-given shortcomings is our goal in the future.

## Figures and Tables

**Figure 1:** PRISMA flow diagram study selection process.

**Table 1:** Search strategy.

1. Amlodipine[Mesh] OR amlodis OR astudal OR norvasc OR istin OR amlor
2. Captopril[Mesh] OR lopirin
3. Enalapril[Mesh] OR renitec OR renitek
4. Felodipine[Mesh] OR felo puren OR felobeta OR felocor OR felodipin
5. Indapamide[Mesh] OR metindamide
6. Losartan[Mesh]
7. Levamlodipine[Supplementary concept]
8. Nitrendipine[Mesh] OR niprina OR nitrendepat OR nitren acis OR nitrendimerck OR nitrendipin
9. Telmisartan[Mesh] OR pritor OR micardis
10. Ramipril[Mesh] OR vesdil OR triatec OR altace OR zabien OR ramace
11. Benazepril[Supplementary concept] OR benazapril
12. Fosinopril[Mesh] OR fosenopril OR fosinil
13. Valsartan[Mesh] OR diovan OR vals
14. Nifedipine[Mesh] OR adalat OR fenigidin
15. Diltiazem[Mesh] OR dilzem OR aldizem
16. Bisoprolol[Mesh]
17. Atenolol[Mesh] OR tenormine
18. Verapamil[Mesh]
19. Hydrochlorothiazide[Mesh] OR HCTZ
20. Acupuncture Therapy[Mesh] OR acupuncture treatment OR therapy, acupuncture OR pharmacoacupuncture OR Acupotom^*∗*^ OR needl^*∗*^
21. OR 1–20
22. Hypertension[Mesh] OR blood pressure, high OR high blood pressure
23. “Drug-related side effects and adverse Reactions”[Mesh] OR “drug related side effects and adverse reactions” OR “side effects of drugs OR drug side effect” OR “adverse drug reaction” OR “reactions, adverse drug” OR “adverse drug event”
24. “Randomized controlled trials as Topic”[Mesh] OR “randomized controlled trial”[Publication type] OR blind OR random^*∗*^
25. 21 AND 22 AND 23 AND 24

## Data Availability

The data used to support the study are included in the paper.

## References

[1] Psaty B. M., Smith N. L., Siscovick D. S., Koepsell T., Weiss T. (1997). Health outcomes associated with antihypertensive therapies used as first-line agents. a systematic review and meta-analysis. *JAMA, the Journal of the American Medical Association*.

[2] Liu D. (2017). Analysis of adverse drug reactions of captopril combined with diuretics in the treatment of hypertension. *Continuing Medical Education in China*.

[3] Kaplan R. C., Psaty B. M., Heckbert S. R., Smith N. L., Lemaitre R. N. (1999). Blood pressure level and incidence of myocardial infarction among patients treated for hypertension. *American Journal of Public Health*.

[4] Chapman A. B., Schwartz G. L., Boerwinkle E., Turner S. T. (2002). Predictors of antihypertensive response to a standard dose of hydrochlorothiazide for essential hypertension. *Kidney International*.

[5] Wu X. (2017). Research progress of acupuncture intervention in prehypertension. *Electronic Journal of clinical medicine literature*.

[6] Wang F. (2017). Comments on the definition of “acupuncture science”. *Chinese Acupuncture & Moxibustion*.

[7] Wang S. (2012). Rational application of antihypertensive combination drugs. *Chinese medical guidelines*.

[8] Qin Y. (2018). Observation and nursing of adverse reactions of antihypertensive drugs in elderly patients. *World latest medical information abstract*.

[9] McDowell S. E., Thomas S. K., Coleman J. J., Aronson J. K., Ferner R. E. (2013). A practical guide to monitoring for adverse drug reactions during antihypertensive drug therapy. *Journal of the Royal Society of Medicine*.

[10] Oertelt-Prigione S., Regitz-Zagrosek V. (2009). Gender aspects in cardiovascular pharmacology. *Journal of Cardiovascular Translational Research*.

[11] Alhawassi T. M., Krass I., Bajorek B. V., Pont L. G. (2014). A systematic review of the prevalence and risk factors for adverse drug reactions in the elderly in the acute care setting. *Clinical Interventions in Aging*.

[12] Higgins J., Deeks J., Higgins J. P. T., Green S. (2008). Selecting studies and collecting data. *Cochrane Handbook of Systematic Reviews of Interventions*.

[13] Moher D., Shamseer L., Clarke M. (2015). Preferred reporting items for systematic review and meta-analysis protocols (PRISMA-P) 2015 statement. *Systematic Reviews*.

[14] Cifu A. S., Davis A. P. (2017). Prevention, detection, evaluation, and management of high blood pressure in adults. *JAMA*.

[15] Lundh A., Gotzsche P. C. (2008). Recommendations by cochrane review groups for assessment of the risk of bias in studies. *BMC Medical Research Methodology*.

[16] Puhan M. A., Schünemann H. J., Murad M. H. (2014). A GRADE Working Group approach for rating the quality of treatment effect estimates from network meta-analysis. *BMJ*.

[17] Jiu-long M. A., Chen Y., Fu X., Xiu-bo S. U. N., Ou L. (2019). Systematic evaluation and meta analysis of adverse. *Practical Pharmacy and Clinical Remedies*.

[18] Neal B., Macmahon S. (1999). The world health organization—International society of hypertension blood pressure lowering treatment trialists’ collaboration: Prospective collaborative overviews of major randomized trials of blood pressure-lowering treatments. *Current Hypertension Reports*.

[19] Ostchega Y., Dillon C. F., Hughes J. P., Carroll M., Yoon S. (2007). Trends in hypertension prevalence, awareness, treatment, and control in older U.S. Adults: data from the national health and nutrition examination survey 1988 to 2004. *Journal of the American Geriatrics Society*.

[20] Düsing R. (2006). Overcoming barriers to effective blood pressure control in patients with hypertension. *Current Medical Research and Opinion*.

[21] Borzecki A. M., Oliveria S. A., Berlowitz D. R. (2005). Barriers to hypertension control. *American Heart Journal*.

[22] Ramli A., Ahmad N. S., Paraidathathu T. (2012). Medication adherence among hypertensive patients of primary health clinics in Malaysia. *Patient Preference and Adherence*.

[23] Holt E. W., Muntner P., Joyce C. J., Webber L., Krousel-Wood M. A. (2010). Health-related quality of life and antihypertensive medication adherence among older adults. *Age and Ageing*.

[24] Wan W., Ma C., Xiong X. (2009). Clinical observation on therapeutic effect of electroacupuncture at Quchi (LI 11) for treatment of essential hypertension. *Chinese Acupuncture & Moxibustion*.

[25] Zhi J., Wang C., Wang Li, Liu Q. (2009). Effect of different quantity of acupuncture stimulation on cervical sympathetic discharge in rats with stress-induced hypertension. *Journal of Traditional Chinese Medicine*.

[26] Esler M. D., Eikelis N., Lambert E., Straznicky N. (2008). Neural mechanisms and management of obesity-related hypertension. *Current Cardiology Reports*.

[27] Huang D., Zhang L. (2010). Effect of needling quchi and zusanli on blood pressure and insulin resistance in spontaneously hypertensive rates. *Journal of Liaoning University of Traditional Chinese Medicine*.

